This article has been retracted.

# Artificial Intelligence Algorithm-Based Analysis of Ultrasonic Imaging Features for Diagnosis of Pregnancy Complicated with Brain Tumor

**DOI:** 10.1155/2021/4022312

**Published:** 2021-11-25

**Authors:** Lin Wu, Donghui Wei, Ning Yang, Hong Lei, Yun Wang

**Affiliations:** ^1^Department of Gynaecology, The Centre Hospital Weinan, Weinan 714000, Shaanxi, China; ^2^Department of Neurosurgery, The Centre Hospital Weinan, Weinan 714000, Shaanxi, China

## Abstract

This research was to explore the accuracy of ultrasonic diagnosis based on artificial intelligence algorithm in the diagnosis of pregnancy complicated with brain tumors. In this study, 18 patients with pregnancy complicated with brain tumor confirmed by pathology were selected as the research object. Ultrasound contrast based on artificial bee colony algorithm was performed and diagnosed by experienced clinicians. Ultrasonic image will be reconstructed by artificial bee colony algorithm to improve its image display ability. The pathological diagnosis will be handed over to the physiological pathology laboratory of the hospital for diagnosis. The doctor's ultrasonic diagnosis results were compared with the pathological diagnosis stage results of patients, and the results were analyzed by statistical analysis to evaluate its diagnostic value. The comparison results showed that the number and classification of benign tumors were the same, while in malignant tumors, the number diagnosis was the same, but there was one patient with diagnostic error in classification. One case of mixed glial neuron tumor was diagnosed as glial neuron tumor, and the diagnostic accuracy was 94.44% and the *K* value was 0.988. The diagnostic results of the two were in excellent agreement. The results show that, in the ultrasonic image diagnosis of patients with brain tumors during pregnancy based on artificial intelligence algorithm, most of them are benign and have obvious symptoms. Ultrasound has a good diagnostic accuracy and can be popularized in clinical diagnosis. The results can provide experimental data for the clinical application of ultrasonic image feature analysis based on artificial intelligence as the diagnosis of pregnancy complicated with brain tumors.

## 1. Introduction

Brain tumors, namely, intracranial tumors, are new organisms directly growing in the brain, including but not limited to new organisms originating in the brain, meninges, nerves, blood vessels, and cerebral appendages or transferred into the brain by other organs and tissues. Brain tumors can be seen in all ages and are most common in 30–50 years old [1]. Clinically, headache, vomiting, visual impairment, mental disorders, unilateral limb sensory abnormalities, hallucinations, hemiplegia or action stumbles, and tinnitus and deafness are caused by increased intracranial pressure and local lesions [2]. Some of its symptoms are similar to those of pregnant women, such as vomiting, headache, and unilateral limb sensory abnormalities, which have caused many inconveniences in the treatment of brain tumors in pregnant women [3, 4]. According to relevant studies, pregnancy whether primary or metastatic brain tumors are rare, which may be due to the reproductive age not the age of multiple brain tumors [5]. Pregnancy itself does not increase the risk of brain tumors, but some patients with brain tumors during pregnancy may have accelerated growth or more obvious symptoms, some of which may be related to the role of sex hormones, especially meningioma and astrocytoma. According to relevant studies, progesterone receptors can be detected in meningiomas, and human astrocytoma cultured in vitro can undergo progesterone accelerated growth [6, 7].

At present, international scholars focus on the treatment of pregnancy complicated with brain tumor. Lynch et al. [8] followed up 6 patients with brain tumors during pregnancy and finally concluded that meningioma is the most common disease type of patients with brain tumors during pregnancy, and pregnancy will aggravate the clinical course of intracranial tumors. Zwinkels et al. [9] followed up the pregnancy of women with glioma during treatment and concluded that low-grade neuroglioma was more common in patients with brain tumors during pregnancy, while high-grade neuroglioma was more likely to be a new phenomenon. Evans et al. [10] found that in a 19-year-old pregnant patient with anaplastic oligodendroglioma during treatment, the doctor stopped using temozolomide and began to track and observe that patient, and the patient finally gave birth smoothly. The doctor concluded that patients with brain tumors should strengthen pregnancy avoidance during chemotherapy to prevent pregnancy from promoting brain tumors.

For brain tumors, due to the lack of understanding of most of them, they lack sufficient understanding of their early symptoms that are considered to be the symptoms of other diseases, thus delaying early diagnosis and treatment. At present, the diagnosis of brain tumors is mainly based on imaging examination, and the common imaging examinations include X-ray film, ultrasonic diagnosis, computed tomography (CT), magnetic resonance imaging (MRI), and pathological examination [11–16].

In recent years, computer-aided diagnosis (CAD) has been widely used in the medical field. The medical influence is analyzed and calculated by computer to improve the image accuracy, which greatly improves the diagnosis efficiency and accuracy. The progress of artificial intelligence makes this technology have a new direction of development, especially the combination of artificial bee colony algorithm and ultrasonic image feature analysis. Artificial bee colony algorithm is often used for reconstruction and analysis of feature parts in similar images, which can greatly improve the ultrasonic image in the exploration of lesions and pathological judgment, but there is no research on this aspect at present. Therefore, the combination of artificial bee colony algorithm and ultrasound image will have a good application prospect in the field of early diagnosis of pregnancy complicated with brain tumor [17, 18].

Due to the existence of pregnancy, the diagnosis and treatment of patients also need to consider the state of the fetus. At present, there is no unified theory to deal with pregnancy complicated with brain tumors. Most of them are individualized, multidepartment comprehensive consideration, and collaborative treatment. The sequence of craniotomy for brain tumors and production operations for children shall be comprehensively considered based on fetal development and brain tumor status. For patients with brain tumor in early pregnancy, it is recommended to stop pregnancy. For patients with benign brain tumors, craniotomy can be performed after full-term production according to the situation. For patients with middle and late stage and large brain tumors, immediate craniotomy is recommended to reduce intracranial pressure [19, 20].

Because the incidence rate of brain tumor is not high in pregnancy, there are few related studies. In this research, artificial bee colony algorithm was innovatively combined with ultrasound image to study the role of this method in the diagnosis of brain tumors during pregnancy, expecting to provide a more effective clinical diagnosis with higher diagnostic efficiency and accuracy. This study will take 18 cases of pregnancy diagnosed with brain tumor in hospital as the research object and use artificial intelligence algorithm to analyze the ultrasonic image characteristics. By comparing with the pathological diagnosis results, we can judge its clinical value in the early diagnosis of pregnancy complicated with brain tumors.

## 2. Research Objects and Methods

### 2.1. Research Object

In this study, 18 pregnant patients with brain tumors in hospital were collected as the research objects, including 23∼33-year-old ones, with an average age of 27.73 ± 4.59 years old. The average gestational week was 28.15 ± 11.65 weeks. There were 16 primipara and 2 multipara women. There were 4 cases in early pregnancy and 14 cases in middle and late pregnancy. This study has been approved by the medical ethics committee of hospital. The patients and their families understood the study and signed the informed consent form.

  Inclusion criteria: (1) patients who have been diagnosed brain tumor during pregnancy; (2) no other tumor metastasis and tissue and organ diseases; (3) the fetus is developing normally
  Exclusion criteria: (1) patients with other serious heart, kidney, liver, and other organ diseases; (2) patients with severe mental illness and unable to communicate normally; (3) family members and patients are reluctant to participate

### 2.2. Diagnosis Scheme

All cases which met the admission requirements were analyzed by ultrasound images based on artificial intelligence algorithm. The instrument used the two-dimensional ultrasound machine, and the probe model was LOGIQ E9,12L. Ultrasonic contrast agent is self-made “lipid fluoride development,” particle size is 1∼5 *μ*m, the main range is 1∼2 *μ*m, and microbubble concentration is 5∼7 × 10^9^ mL. The patient was bedridden, and the probe was wrapped by sterile endoscopic package with a small amount of saline injected. The saline was used as the oral contact agent for skull flap creation, and the dura mater or brain surface was examined by the operator along the coronal, sagittal, horizontal, and surface. The examination image results were analyzed based on the characteristics of artificial intelligence algorithm and were operated by two physicians who did not know the pathological examination results. The examination results were given, respectively. For the conflicting results, the unified results were discussed by two physicians.

### 2.3. Ultrasonic Imaging Based on Artificial Intelligence Algorithm

Based on the artificial intelligence algorithm, this study will use the image reconstruction based on the artificial bee colony (ABC) algorithm commonly used in medical images to analyze the characteristics of image results. Image reconstruction based on artificial bee colony can reconstruct the image. Compared with traditional image segmentation, artificial bee colony optimization can take tumor eigenvalues as classification samples and reduce feature dimensions. In reducing support vector machine (SVM), it greatly improves the accuracy of the image for key parts and the embodiment of small tissue parts. It is widely used in medical imaging.

Firstly, the texture feature of tumor needs to be extracted. According to the texture feature value proposed by Chen et al. [21] as the regularized autocorrelation function, it is assumed that the custom pixel (*i*, *t*) and pixel (*i*+Δ*p*, *t*+Δ*q*) in an image with a size of *P* × *Q* are regularized as *ν*(Δ*p*, Δ*q*)=*A*(Δ*p*, Δ*q*)/*A*(0,0).

(1) $$\begin{array}{c} A\left(\Delta p,\Delta q\right)=\frac{1}{\left(p-\Delta p\right)\left(q-\Delta q\right)}\overset{p-\Delta p-1}{\underset{x=0}{\sum }}\overset{q-\Delta q-1}{\underset{y=0}{\sum }}f\left(x,y\right)f\left(x+\Delta p,y+\Delta q\right). \end{array}$$

In order to eliminate the influence of image brightness factors, the average brightness value $\bar{f}$ is added to

(2) $$\begin{array}{c} A^{1}\left(\Delta p,\Delta q\right)=\frac{1}{\left(p-\Delta p\right)\left(q-\Delta q\right)}\overset{p-\Delta p-1}{\underset{x=0}{\sum }}\overset{q-\Delta q-1}{\underset{y=0}{\sum }}\left(f\left(x,y\right)-\bar{f}\right)\left(f\left(x+\Delta p,y+\Delta q\right)-\bar{f}\right). \end{array}$$

Therefore, the texture eigenvalue of brain tumor is defined as

(3) $$\begin{array}{c} \nu^{1}\left(\Delta p,\Delta q\right)=\frac{A^{1}\left(\Delta p,\Delta q\right)}{A^{1}\left(0,0\right)}. \end{array}$$

For the tumor contour, its geometric characteristics are defined as six types in this study, namely, shape coefficient *A*, roundness *B*, aspect ratio *C*, convex surface *D*, volume *E*, and range *F*, as shown in equations (4)–(9).

(4) $$\begin{array}{c} A=\frac{4\pi \cdot M}{Z^{2}}, \end{array}$$

(5) $$\begin{array}{c} B=\frac{4\pi \cdot M}{\pi \cdot J_{\text{Max}}^{2}}, \end{array}$$

(6) $$\begin{array}{c} C=\frac{J_{\text{Max}}}{J_{\text{Min}}}\cdot B, \end{array}$$

(7) $$\begin{array}{c} D=\frac{T}{Z}, \end{array}$$

(8) $$\begin{array}{c} E=\frac{N-M}{\sum_{i=1}^{n}N_{i}-\left(M_{i}/n\right)}, \end{array}$$

(9) $$\begin{array}{c} F=\frac{M}{K}. \end{array}$$

Here, *M* is area, *Z* is perimeter, *J* is diameter, *T* is perimeter of polygon surrounding tumor, *N* is area of the smallest polygon surrounding the tumor, *K* is area of the smallest rectangle surrounding the tumor, and *n* is natural number. Schematic diagram of geometric parameters is shown in Figure 1.

SVM is a common method to solve data classification analysis. It uses the optimal hyperplane in data classification and processes two-dimensional linear nonseparable samples by high-dimensional mapping of kernel function, so as to obtain the global optimal solution.

The image reconstruction of the artificial bee colony algorithm proposed in this study mainly includes four elements: food source (problem to be solved), hired bee, reconnaissance bee, and following bee, and two behavior modes: searching food source and abandoning food source. Firstly, the artificial bee colony algorithm randomly generates *N* solutions (food source). *x*_*q*_(*q*=1,2,…, *N*) is a vector of the problem to be solved or data classification size *D*. All solutions are searched by the bee colony until the maximum search times (*K*) is reached. The hired bee records the corresponding food source and looks for a new food source near the food source, so that a better food source can be found to replace the original food source. Each time the search is completed, the hired bee returns to the nest and transmits the location, distance, and quantity of the food source to the follower bee. The follower bee selects the food source according to the obtained information. The higher the quality of the food source, and the more likely it is to be selected. The selected probability *Z* can be solved according to

(10) $$\begin{array}{c} Z_{q}=\frac{{\text{fit}}_{q}}{\sum_{n-1}^{N}{\text{fit}}_{n}}, \end{array}$$

where fit_*q*_ represents the appropriate value of the *q*th solution. The search range of hired bee and follower bee is

(11) $$\begin{array}{c} W_{it}=Y_{it}+R_{it}\left(Y_{it}-Y_{ut}\right), \end{array}$$

which is a random parameter, but the two parameters are not equal. *R*_*it*_ is a random variable between [−1,1], and *Y*_*it*_ is a variable that controls the scope of searching food source.

The specific process of artificial bee colony algorithm is shown in Figure 2.

The brain tumor eigenvalues and SVM parameters were screened according to the artificial bee colony algorithm. Each bee contains the eigenvalues and SVM parameters to be filtered. SVM is used to calculate the accuracy after filtering and then sent to ABC algorithm. ABC algorithm performs operation again until the upper limit of operation times is reached.

### 2.4. Simulation Experiment

To evaluate the effect of image reconstruction, the commonly indexes are used to calculate the mean square error (MSE) and peak signal-to-noise ratio (PSNR) of the reconstructed image and test image. The calculation equation of MSE is as follows:

(12) $$\begin{array}{c} \text{mean square error}=\frac{1}{L\times W}\sum_{i=1}^{L}\sum_{j=1}^{W}{\left(C_{1}\left(i,j\right)-C_{2}\left(i,j\right)\right)}^{2}. \end{array}$$

*C*_1_ represents the reconstructed image, *C*_2_ is the test image, *L* is the image length, and *W* is the image width. The smaller the MSE, the finer the reconstructed image.

PSNR is the most commonly used evaluation index in the field of image processing, and its equation is as follows:

(13) $$\begin{array}{c} \text{peak signal}‐\text{to}‐\text{noise ratio}=10\;{\text{Log}}_{10}\left(\frac{{\left(2^{b}-1\right)}^{2}}{\text{MSE}}\right), \end{array}$$

where *b* represents the number of bits per pixel. The greater the PSNR, the higher the quality of image reconstruction.

Data samples are selected and divided into image block of 8 × 8, 10,000 of which are selected as training samples to construct the training data of artificial bee colony learning model and reconstruct the image after feature analysis. K-singular value decomposition (K-SVD) algorithm and stacked autoencoder (SAE) are selected for data analysis and image reconstruction and compared with the reconstructed image of artificial bee colony algorithm [22, 23]. K-SVD is a kind of classical dictionary training algorithm, but compared with general dictionary training, it only updates one column of data each time, so it is often used for image compression sensing. SAE is a kind of unsupervised algorithm, which is mainly used for the restoration perception of the original image. These two algorithms are used as a comparison algorithm to compare the image reconstruction ability of the artificial bee colony algorithm selected in this paper.

The experimental environment is win10 system, CPU: Intel(R)Celeron(R)CPU1007U@1.50 GHz, MATLAB platform.

### 2.5. Statistical Study

In this study, Medcalc version analysis statistics software is used for data processing, Kappa consistency test is used for correlation, and the test level is *∝* = 0.05. The reference evaluation of *K* (Kappa) value is as follows: *K* ≤ 0.40, poor diagnostic consistency; 0.40 < *K* ≤ 0.75, good diagnostic consistency; 0.75 < *K* ≤ 1, the diagnostic consistency is excellent.

## 3. Results

### 3.1. Algorithm Simulation Results

Figure 3 shows the input test sample.

The test chart is divided into image block of 8 × 8. The reconstruction results of the three algorithm models are shown in Figure 4.

Figure 4(a) is an SAE reconstructed image.  Figure 4(b) is a reconstructed image of K-SVD.  Figure 4(c) is an image reconstructed by artificial bee colony algorithm. The comparison between the corresponding PSNR and MSE is shown in Figure 5.

Through the comparison of PSNR and MSE of SAE reconstructed image, K-SVD reconstructed image, and artificial bee colony algorithm reconstructed image, it shows that the image reconstruction effect under the artificial bee colony algorithm model is significantly better than SAE reconstruction and KAVD reconstruction. Experiments show that the artificial bee colony algorithm has a good performance in tumor image reconstruction.

### 3.2. Comparison of Diagnostic Results of Pregnancy Complicated with Brain Tumor

After clinical diagnosis, 11 of the 18 patients showed headache, nausea, and vomiting, accounting for 61.11%. The headache was mainly local or whole head pain, intermittent or persistent, and 5 cases (45.45%) showed progressive aggravation. Three patients showed hearing loss, tinnitus, and visual impairment, accounting for 16.67%. Two patients had unilateral limb weakness, accounting for 18.18%. Two patients showed unilateral limb convulsion, accounting for 18.18%. The specific proportion is shown in Figure 6.

Pathological diagnosis showed that there were 5 malignant tumors in 18 patients, including 1 glioblastoma, 2 mixed glioneuronal tumors, 1 astrocytoma, and 1 oligodendroglioma. There were 13 benign tumors, including 6 benign meningiomas, 4 neurofibromas, and 3 acoustic schwannomas.

According to the ultrasonic image characteristics of artificial bee colony algorithm, 5 cases of malignant tumors and 13 cases of benign tumors were diagnosed in 18 patients, which was consistent with the pathological diagnosis. However, there are still errors in the diagnosis of specific tumor types. 5 cases of malignant tumors were diagnosed, including 1 case of glioblastoma, 1 case of mixed glioblastoma, 1 case of ganglioglioma, 1 case of astrocytoma, and 1 case of oligodendroglioma. There were 13 cases of benign tumors, including 6 cases of benign meningioma, 4 cases of neurofibroma, and 3 cases of acoustic schwannoma.

According to the comparative analysis of the ultrasonic image characteristics of artificial bee colony algorithm and the pathological diagnosis in Figure 7, the diagnosis results of benign tumors are consistent, while in malignant tumors, there is one patient with wrong diagnosis, which may be caused by the fact that the ultrasonic images of mixed glial neuron tumors and glial neuron tumors are very similar, and the ultrasonic images are not clearly displayed, but the results are still very similar, with an accuracy rate of 94.44%. After calculation, *K* = 0.988, the diagnostic results of the two methods are in excellent agreement.

### 3.3. Ultrasonic Feature Analysis Image

Figure 8 shows the characteristic analysis image of contrast-enhanced ultrasound for glioma.

## 4. Discussion

Due to its unique physiological factors during pregnancy, its diagnosis and treatment are affected and restricted by more factors. According to relevant studies, most of the pregnancy associated tumors are benign, malignant tumors are rare, and they are more common in older pregnant women. Especially with the opening of the three-child policy, the pregnant age of pregnant women continues to rise, which may further improve the probability of tumor during pregnancy. In order to ensure the life safety of pregnant women and children, early diagnosis, early detection, and early treatment are the best way to effectively reduce the harm of tumor.

Firstly, the ultrasonic image based on artificial intelligence algorithm is verified by experiments. In this study, the artificial bee colony algorithm is used to reconstruct the ultrasonic image to improve the accuracy of the image. It can clearly image small tissues, which is mainly reflected. Through verification experiments, it is confirmed that the artificial bee colony algorithm has better improvement in image accuracy than other image reconstruction methods.

In this study, 18 patients in hospital were selected as the research object, and ultrasound images based on artificial intelligence algorithm were carried out, and professional doctors were invited for diagnosis. According to the comparison between the diagnostic results of ultrasound images based on artificial bee colony algorithm and pathological diagnosis results of pregnant patients with brain tumor, only 1 case was misdiagnosed, and the other cases were consistent with pathological diagnosis results, which may be related to the fact that the ultrasound images of mixed glial neuron tumor and glial neuron tumor are very similar and the ultrasound images are not clear.

In this study, it is determined that ultrasound images based on artificial intelligence algorithm play a positive role in the analysis of pregnancy complicated with brain tumors, especially in the more prominent and clear display of blood vessels, tissues, lesions, and other tissue parts, and play a positive auxiliary role in the diagnosis of pregnancy brain tumors. In addition, because of its clear presentation of the lesion tissue, it can also be used as an imaging guidance scheme for the comparison of operation and prognosis recovery and secondary operation and plays a great role in the preoperative and prognosis of patients.

Hu et al. [24] by using an algorithm based on fuzzy system for brain tumor medical image processing and comparing the results with a variety of artificial intelligence algorithms, found that using this algorithm can be faster and more stable access to quality medical imaging, and the precision of the image is much higher than other algorithms processing results. Latifoğlu [25] proposed an artificial bee colony algorithm to optimize the digital image denoising of ultrasonic images and tested multiple ultrasonic images at the same time. The results showed that this method could effectively eliminate the noise in the test image. Wu et al. [26] designed an artificial bee colony algorithm for processing Doppler ultrasound images, which can greatly improve the quality of ultrasound images, reduce image noise and greatly improve the clinical diagnosis ability of diseases.

## 5. Conclusion

In this study, 18 patients with pregnancy complicated with brain tumor were selected as the research object. The ultrasonic image characteristics based on artificial intelligence were analyzed and compared with the results of pathological examination. The results showed that there was no significant difference between the results of ultrasonic imaging diagnosis of pregnancy complicated with brain tumor based on artificial intelligence and pathological examination. It is proved that this detection method can be used in the clinical diagnosis of pregnancy complicated with brain tumor, which is worthy of popularization. Because there are few patients with pregnancy complicated with brain tumors, it is difficult to select a larger number of studies, which may produce some errors in the results. It is expected that relevant organizations or teams can select more patients for research in the future. At present, there are few studies on pregnancy complicated with brain tumors. The study in this paper proved the clinical value of artificial intelligence algorithm feature analysis in the diagnosis of pregnancy with brain tumor, provided certain clinical data for clinical diagnosis of pregnancy with brain tumor and provided certain research direction for future research of other organizations or teams.

## Figures and Tables

**Figure 1:** Schematic diagram of geometric parameters (*A* is the maximum diameter, *B* is the minimum diameter, *C* is the smallest polygon surrounding the tumor, and *D* is the smallest rectangle surrounding the tumor).

**Figure 2:** Flow chart of the artificial bee colony algorithm.

**Figure 3:** Test diagram.

**Figure 4:** Reconstructed image results.

**Figure 5:** Comparison of simulation results of three reconstruction methods (compared with ABC algorithm, ^*∗*^*P* < 0.05).

**Figure 6:** Proportion of clinical diagnosis.

**Figure 7:** Analysis of characteristics of ultrasonic imaging compared with pathology results (in the figure, (a) is the diagnostic classification of malignant tumors and (b) is the diagnostic classification of benign tumors).

**Figure 8:** Contrast-enhanced ultrasound analysis of glioma features.

## Data Availability

The data used to support the findings of this study are available from the corresponding author upon request.
